# Meta-Analysis on the Improvement of Symptoms and Prognosis of Gastrointestinal Tumors Based on Medical Care and Exercise Intervention

This article has been retracted.

**DOI:** 10.1155/2021/5407664

**Published:** 2021-11-12

**Authors:** Qiqi Le, Chengyan Wang, Qi Shi

**Affiliations:** ^1^Rehabilitation Department, Songnan Community Health Service Center, Shanghai 200441, China; ^2^Oncology Department, Yueyang Hospital of Integrated Traditional Chinese and Western Medicine, Shanghai University of Traditional Chinese Medicine, Shanghai 200437, China; ^3^Oncology Department, Shanghai Municipal Hospital of Traditional Chinese Medicine, Shanghai University of Traditional Chinese Medicine, Shanghai 200071, China

## Abstract

Gastric cancer is a malignant tumor that originates from the epithelium of the gastric mucosa. It is the result of a combination of multiple factors, but the current research has not yet clarified its pathogenesis, so further research and exploration are needed. This article is mainly based on the meta-analysis of the improvement of gastrointestinal tumor-related symptoms and prognosis based on medical care and exercise intervention. The control group followed routine care after enrollment. In addition to routine care, patients in the intervention group exercised through assessment, formulation of exercise prescriptions, implementation of supervision, and adjustment. By viewing the subjects' physical examination reports, determine their blood routine, urine routine, blood lipids, blood sugar, liver and kidney function, and electrocardiogram examination. In this experiment, dual-contrast ultrasound in each T staging was greater than 0.8, indicating that the diagnostic method is very accurate in the preoperative diagnosis of gastric cancer T staging. The results show that exercise intervention can improve the pain of patients with gastrointestinal tumors after chemotherapy, relieve cancer-induced fatigue, and improve the quality of life.

## 1. Introduction

Surgery is still the main treatment for gastrointestinal tumors. Due to the time-consuming, difficult, and frequent changes of the original anatomical structure, patients have a longer postoperative hospital stay and slower prognosis. With the advancement of the concept of accelerated rehabilitation, a series of optimization measures in the perioperative period are gradually improved, but patients still generally complain of fatigue during hospitalization. Moreover, the parents of the “single generation” have also entered the advanced age group, and the burden of the “single generation” in the society on their parents' old-age care is also very huge. As the ratio of patients to doctors and nurses increases, the quality of patient care is also declining.

The malignant process of gastrointestinal tumors is a complex, multistage, and dynamic process. For the diagnosis of gastrointestinal stromal tumors, the computer-aided detection of lymph nodes near the stomach is even more important, because the morphological changes and metastasis of gastric lymph nodes are the wind vane for doctors to diagnose gastrointestinal stromal tumors. Lymph node analysis near the focus can help doctors more accurately determine the patient's lymph node staging, predict its metastasis mechanism, and determine future treatment options, which can strive for a greater survival rate for patients.

Before implementing exercise prescriptions for cancer treatment patients, the pros and cons should be evaluated in advance, including short-term and long-term health risks. When the benefits of exercise outweigh the harms of no exercise, exercise intervention can be chosen to reduce CRF. Tryggestad et al. believe that in recent years, with more and more institutions implementing intensity-modulated proton therapy (IMPT), proton beam radiotherapy (RT) has been rapidly applied in the treatment of gastrointestinal malignancies. Although their research has certain reference value, it lacks a specific implementation process [1]. Pidkovka et al. believe that targeted therapy has changed the treatment model for diseases, but the clinical effect on gastrointestinal malignancies is relatively low. Although their research has a positive effect on the follow-up treatment of patients, it lacks necessary experimental data [2]. Feng et al. believe that the nonopioid analgesic Analgin is used to treat acute and chronic pain and fever. Although their research is relatively comprehensive, some of the content is inaccurate [3].

From the perspective of improving exercise compliance, this research proposes a design method for a personalized exercise plan based on behavior change theory. This study compared the efficacy and safety of different physical interventions (IPC alone or combined with GCS) in preventing DVT during gastrointestinal tumor surgery and explored more effective measures to prevent deep vein thrombosis during gastrointestinal tumor surgery. Intraoperative prevention of DVT provides practical application value.

## 2. Exercise Intervention and Gastrointestinal Tumors

### 2.1. Healthcare

Assuming that the random variable *X* obeys the logistic distribution, the cumulative distribution function of *X* is as follows [4, 5]:

(1) $$\begin{array}{c} F\left(x\right)=\frac{1}{1+\exp\left(-\left(x-\mu \right)/\gamma \right)},\;x\in R. \end{array}$$

The probability density function of *X* is as follows:

(2) $$\begin{array}{c} F\left(x\right)=\frac{\exp\left(-\left(x-\mu \right)/\gamma \right)}{\gamma {\left(1+\exp\left(-\left(x-\mu \right)/\gamma \right)\right)}^{2}},\;x\in R. \end{array}$$

Among them, *μ* is the position parameter, and *γ* is the shape parameter [6].

Generally, maximum likelihood estimation is used to solve the estimated parameters of the regression model. Here, suppose

(3) $$\begin{array}{c} P\left(Y=1|X=x\right)=\pi \left(x\right). \end{array}$$

Then,

(4) $$\begin{array}{c} P\left(Y=1|X=x\right)=\pi \left(x\right). \end{array}$$

For the training dataset of *n* sample points, the likelihood function is [7]

(5) $$\begin{array}{c} L\left(w\right)=\prod_{i=1}^{n}{\left[\pi \left(x_{i}\right)\right]}^{y_{i}}{\left[1-\pi \left(x_{i}\right)\right]}^{1-y_{i}}. \end{array}$$

Therefore, the log likelihood function is [8]

(6) $$\begin{array}{c} l\left(w\right)=\ln\left(L\left(w\right)\right)=\sum_{i=1}^{n}\left[y_{i}\left(w\cdot x_{i}\right)-\ln\left(1+\exp\left(w\cdot x_{i}\right)\right)\right]. \end{array}$$

At this time, the estimated binomial regression model is [9]

(7) $$\begin{array}{c} P\left(Y=1|x\right)=\frac{\exp\left(\hat{w}\cdot x\right)}{1+\exp\left(\hat{w}\cdot x\right)},\\ P\left(Y=0|x\right)=\frac{1}{1+\exp\left(\hat{w}\cdot x\right)}. \end{array}$$

For a given training dataset,

(8) $$\begin{array}{c} T=\left\{\left(x_{1},y_{1}\right),\left(x_{2},y_{2}\right),\ldots ,\left(x_{n},y_{n}\right)\right\}. \end{array}$$

Among them, each sample point is composed of instance *X* and label *Y*, with instance *X*=(*x*^(1)^, *x*^(2)^,…,*x*^(*m*)^)^*T*^ ∈ *R*^*m*^ and label *Y* ∈ {−1,1} [10, 11].

The empirical risk of model *f*(*x*, *w*) is expressed as

(9) $$\begin{array}{c} R_{\text{emp}}\left(f\right)=\frac{1}{n}\sum_{i=1}^{n}l\left(y_{i},f\left(x_{i},\omega \right)\right). \end{array}$$

Among them, *ω* is the generalized parameter of the model, and *l*(·) is the loss function [12].

The covariance matrix of a single event for each type of signal is as follows [13]:

(10) $$\begin{array}{c} C=\frac{E_{N*T}*E_{N*T}}{\text{trace}\left(E_{N*T}*E_{N*T}\right)}. \end{array}$$

Among them, *E*_*N∗T*_ represents the signal matrix of each event, *N* represents the number of channels of the EEG signal, *T* represents the number of sample points of the EEG signal of each event, *i* represents the class label of the motor imaging task, and trace(*X*) represents all the diagonal elements of the matrix *X* are summed [14].

*x* and *y* represent two random variables, respectively, and their mutual information *I*(*x*; *y*) is obtained by their probability density functions *p*(*x*), *p*(*y*), and *p*(*x*, *y*) [15]:

(11) $$\begin{array}{c} I\left(x;y\right)=\oint p\left(x,y\right)\log\frac{p\left(x,y\right)}{p\left(x\right)p\left(y\right)}\text{d}\varphi , \end{array}$$

where *x* is a discrete feature vector, *y* is a discrete feature vector or class label, and *p*(*x*) and *p*(*y*) represent edge probability functions. Among them, 0 means completely independent and 1 means completely related [16].

In order to obtain the EEG signal features that are highly related to the category, the features are selected in the optimal feature set according to their correlation from largest to smallest using the method of maximum correlation [17].

(12) $$\begin{array}{c} \max\;D\left(f,c\right),\\ D=S\frac{1}{{\left|S\right|}^{2}}\sum_{f_{i}\in s}I\left(f_{i};f_{j}\right). \end{array}$$

Among them, *f*_*i*_ refers to the *i*-th feature, and *c* refers to the class label [18].

Assuming that there are two random time series *X* and *Y,* respectively, the joint entropy between the two is defined as

(13) $$\begin{array}{c} H\left(X,Y\right)=-\sum_{x}\sum_{y}P\left(x,y\right)\log_{2}\left[P\left(x,y\right)\right]. \end{array}$$

Among them, *x* and *y* are the data values in the random sequence *X* and *Y,* respectively, and *P*(*x*, *y*) represents the joint probability value of *x* and *y* together [19, 20].

In order to make the communication protocol of the system architecture in this design independent, a simple communication protocol is designed in the application layer, that is, an abstraction layer is inserted between the sensor device and the mobile monitoring center. The reason for adopting this design is that there is no current standard that meets the demand on the market. Although people have done a lot of work in realizing standardization, realizing standardization in the field of body sensor networks is still in the development stage. Therefore, setting up the communication protocol for medical equipment in this design can meet the design requirements of this platform and provide an overall solution to the potential future needs of the platform [21, 22].

### 2.2. Tumors of the Digestive Tract

The influence of digestive tract microorganisms on cancer treatment is shown as Figure 1. Since the size of the stomach CT image is 512 × 512, and the stomach parenchyma is always in the middle part of the image, the migration of tumor cells from the primary tumor to specific tissues and organs to form metastases requires a series of biological processes. Tumor-associated macrophages are derived from mature monocytes in peripheral blood and undergo morphological and functional changes under the effects of chemokines and cytokines secreted by tumor cells, tumor stromal cells, and immune cells, and under the influence of different tissue environments in the body, many immune cells will be produced around tumor cells, which can secrete a variety of cytokines, which are potential targets for immune regulation and tumor immunotherapy [23].

### 2.3. Exercise Intervention

Exercise intervention is a nonsurgical treatment method, which aims to improve people's bad behaviors through scientific and reasonable guidance arrangements for the patient's exercise mode, type, time period, and frequency, so as to achieve the purpose of treating or preventing diseases. The basic principles of sports intervention are safety, effectiveness, accuracy, and practicality. Exercise intervention can affect the behavior, consciousness, and social relations of people with different cultures, lifestyles, and economic conditions, which can improve the group's pressure coping style and psychological endurance. At present, exercise intervention is widely used in clinics, especially in chronic diseases and mental diseases. It can be seen that participating in physical exercise three to four times a week is the most suitable exercise frequency. Considering the accumulation of exercise effects, the interval of exercise intervention should not exceed three days. Therefore, when the total amount of exercise is determined, the exercise intensity and exercise time are inversely proportional, that is, the exercise time should be set shorter when the exercise time intensity is high, and the exercise time should be set longer when the exercise intensity is low.

## 3. Exercise Intervention to Improve the Symptoms and Prognosis of Gastrointestinal Tumors

### 3.1. Subjects

In this paper, convenience sampling was used to select 60 eligible patients with gastrointestinal cancer chemotherapy. In this study, 29 males and 31 females were enrolled in the group, with an average age of 42 ± 11.5, including 18 gastric cancer, 6 esophageal cancer, 15 colon cancer, and 21 rectal cancer patients.

### 3.2. Development and Implementation of Sports Interventions

After joining the control group, routine care was followed, the nutritional status of patients was comprehensively evaluated, malnutrition and anemia were corrected, blood routine and liver function were checked, and corresponding measures were taken when abnormalities occurred, chemotherapy-related knowledge was educated, nutrition was supplemented, and daily activities were encouraged. After enrolling patients in the intervention group, in addition to routine care, exercise was carried out through assessment, formulation of exercise prescriptions, implementation of supervision, and adjustment, as follows. Assessment: patient age, heart rate, and blood pressure. Formulating exercise prescription: exercise frequency is 3∼4 times a week, exercise is 20∼30 minutes each time, and the heart rate during exercise reaches 65%∼85% of the maximum heart rate. Exercise form: aerobic exercises such as brisk walking, up and down stairs, badminton, and swimming were chosen according to the patient's preferences. Instructing patients to exercise: patients were instructed to self-test their pulses when they are admitted to the hospital for the first time, a mobile phone APP was installed to detect heart rate, 5–10 minutes of warm-up activities were performed before exercise and 5–10 minutes after exercise. Supervision: patients were instructed to use exercise diaries to record their exercise status and we call back to monitor the implementation status after discharge from the hospital and ask about the guidance exercise status every time they return to the hospital for chemotherapy.

### 3.3. Blood Test

On the second day of the study subject's admission to the hospital for routine blood sampling, the blood sample was collected with an EDTA tube to reduce the patient's repeated blood sampling invasive operation; after collecting the blood, the blood sample was put on the centrifuge and it was set to 2500 rpm for 10 minutes. After centrifugation, the serum was separated from the red blood cells quickly and carefully to avoid hemolysis; after obtaining the serum, the serum specimens were stored in a refrigerator at −70°C. After all blood samples are collected, they will be sent to the testing center for testing. The principle of blood testing: the double-antibody one-step sandwich enzyme-linked immunosorbent assay is used to measure the changes of cytokine interleukin-1*β*, interleukin-6 content, and tumor necrosis factor-*α* in the patient's serum. Routine blood drawn before and after radiotherapy is routinely sent to the laboratory to test the neutrophil count value.

### 3.4. Inflammation Indicators

At 8 o'clock in the morning of the test day, the subjects went to the outpatient building of the Institute of Sports Medicine of the State General Administration of Sports on an empty stomach. The test indicators are interleukin-6 (IL-6) and tumor necrosis factor (TNF-*α*), and the test method is enzyme-linked immunoassay.

### 3.5. Health Screening before Exercise

All subjects were screened through questionnaires, including current medical history, family history, disease history, history of tobacco and alcohol, history of medication, history of allergies, physical activity, or exercise habits. Determine the subjects' blood routine, urine routine, blood lipids, blood sugar, liver and kidney function, electrocardiogram by calling the physical examination report.

### 3.6. Health Fitness Test and Evaluation

Test items include height (cm), weight (kg), vital capacity (ml), step index, grip strength (kg), sitting forward bending (cm), standing on one foot with closed eyes (seconds), reaction time (seconds), exercise time (seconds), 1 minute heart rate (times), 2 minutes heart rate (times), and 3 minutes heart rate (times). A full set of “Jianmin Type 4 National Fitness Test” equipment was used to test, and Inbody370 body composition tester was used to complete the BMI and body fat percentage (%).

### 3.7. Statistical Processing

Stata 13.0 and Microsoft Excel 2010 were used for analysis. For continuous data, the total mean weighted by the sample size and the standard deviation of the sample mean (or median) are calculated, and the categorical data are expressed as percentage. The heterogeneity test uses X2 and I2 to evaluate; *P* > 0.05 or I2 < 50% indicates that the heterogeneity is low. The comparative study of the two measures used HRs and its 95% confidence interval (95% CI) combined evaluation; *P* < 0.05 considered the difference to be statistically significant.

## 4. Results and Discussion

The influence of time and intervention factors on the objective nutritional indicators of the two groups of patients is shown in Table 1. A two-factor three-level repeated-measurement analysis of variance method was used to compare the differences between the two groups of objective nutritional indicators at 3 time points (before intervention, 21 days after intervention, and one month after follow-up). The results showed that the objective indicators of the two groups of patients were consistent. The difference in main effects of HB and ALB time, the difference in main effects of intervention, and the difference in interaction between intervention factors and time factors were all statistically significant (*P* < 0.05), indicating that the HB and ALB values of the two groups of patients vary with each other without considering the intervention factors. Time changes and changes; regardless of the time factor, the HB and ALB values of different intervention levels are different; at the same time, the change trend is different at different time points under different intervention levels.

The performance evaluation of the AdaBoost diagnostic model is shown in Table 2. In the end, it can be concluded that for the case dataset 1, the average correct rate of the AdaBoost classification diagnosis model is 89.91%, and the average *F*1 score is 77.53%. The diagnosis effect of the model is better.

The symptom cluster of patients with gastrointestinal cancer during chemotherapy is shown as Figure 2. The symptoms with factor load ≥0.4 were included in the symptom group. In this paper, 5 symptom groups were extracted, and the cumulative variance contribution rate was 68.381%. There are still 23.7% of patients who do not exercise normally, and the duration of exercise is half an hour or more of the patients accounted for 59.8%, and the remaining 40.2% of patients had insufficient exercise time. Therefore, strengthening the specific guidance of patients' exercise and relaxation, helping patients to formulate their own relaxation and exercise plan, is of great significance to promoting their symptom coping and physical recovery.

Table 3 shows the combined effect size of dual-contrast ultrasound in the diagnosis of T staging of gastric cancer. Sensitivity analysis is used to detect whether a certain study has a decisive significance to the combined total results. Generally, after excluding each study one by one, observe whether the heterogeneity and combined diagnostic indicators have changed, so as to analyze the stability of the results of this study. In this experiment, dual-contrast ultrasound in each T staging was greater than 0.8, indicating that the diagnostic method is very accurate in the preoperative diagnosis of gastric cancer T staging.

Single factor repeated measures analysis of variance was used to determine the effect of 6-week exercise intervention on subjects' CRF. The comparison of the BFI scores of the two groups of patients is shown as Figure 3. The difference is that the fatigue of the 4th and 6th courses of the experimental group is better than that of the control group, the fatigue of the 6th course of the experimental group is better than the 4th course, and the fatigue of the 4th course of the control group is heavier than the first course.

The ultrasound appearance of gastrointestinal tumors is shown in Figure 4. Different types of stomach nodules were unfold into a time series, and the smoothness of the time series was compared to easily distinguish the difference between no sign, leaf sign, and glitch sign. However, the time series of gastric nodules with no signs and lobulated signs are relatively smooth and cannot be distinguished effectively. The recursive graph algorithm comprehensively considers the chaos, nonstationary, and periodicity of the gastric nodules boundary, and the difference between the common sign and the lobular sign is obvious, so as to achieve the effect of detecting gastric nodules. At the same time, the algorithm in this paper has high specificity and low misdiagnosis rate, which avoids the interference of nonnodules to the doctor's diagnosis to a certain extent and saves the doctor's diagnosis time. The algorithm is stable and reliable, does not depend on the overall gray value of the image, and has strong adaptability, which is conducive to the actual clinical application of gastric CAD.

Table 4 shows the comparison of lower extremity vein diameter (mm) of the two groups of patients before and after surgery. As a result, the preoperative independent sample *t* test value of the two groups was *t* = −0.847, *P*=0.399 > 0.05; the diameter of the common femoral vein *t* = 1.8, *P*=0.07 > 0.05; the deep femoral vein *t* = 1.205, *P*=0.231 > 0.05. In the IPC group, the diameter of the vein before and after the operation was paired with *t* test. The diameter of the popliteal vein *t* = −1.769, *P*=0.083 > 0.05; the difference was not statistically significant. In the IPC + GCS group, a paired *t*-test was performed on the diameter of the vein before and after the operation. The diameter of the external iliac vein was *t* = −1.096, *P*=0.279 > 0.05.

The comparison of the weight changes of patients with different nutritional status 48 hours after admission and 7 days after operation is shown in Figure 5. At the time of admission, the weight of patients with nutritional status of SGA A was 67.40 ± 9.69 kg, SGA B was 0.60.75 ± 9.78 kg, and SGA C was 49.60 ± 8.18 kg. After analysis of variance and LSD test, the difference in preoperative weight of the three groups of patients was as follows: statistically significant, *P* < 0.01. At 7 days postoperatively, the body weights of the SGAA, SGAB, and SGAC groups were 65.11 ± 9.40 kg, 58.34 ± 9.25 kg, and 47.85 ± 7.09 kg, respectively. After analysis of variance and LSD test, the difference in postoperative body weight of the three groups was statistically significant, *P* < 0.01. During the hospitalization, the patient did not gain weight, among them, the weight of the SGAA group was reduced by 2.29 ± 1.71 kg, the SGAB group was reduced by 2.41 ± 2.06 kg, and the SGAC group was reduced by 1.95 ± 1.99 kg. After the analysis of variance, there was no difference in the perioperative weight loss of the three groups. *P* > 0.05 was statistically significant.

The relationship between EphA1 mRNA expression and clinicopathological indicators is shown in Figure 6. The PCR product of EphA1 mRNA is a 127 bp fragment. The expression of EphA1 was detected in 65 patients with gastric cancer, but there are differences in expression, that is, there are high expression, low expression, and normal expression. EphA1 expression in cancer cells was upregulated in 19 cases (29.2%) and downregulated in 20 cases (30.8%), and the remaining 26 cases (40.0%) had no difference in expression between the cancer cells and normal mucosal cells.

Table 5 shows the comparison of the degree of total fatigue and the degree of each dimension before and after the exercise prescription intervention. The exercise intervention prescription adopted in this study can well improve the fatigue of gastric cancer patients.

The RT-PCR method to detect the relative expression of PTEN and Notch1 mRNA when doxorubicin interferes with gastric cancer cell BGC-823 at different time gradients is shown as Figure 7. When gastric cancer cells were disturbed for 3, 6, and 12 hours, the cell survival rates were 58.46%, 84.93%, and 46.27%, respectively, which decreased in a time-dependent manner, and compared with the control group at 0 h, the difference was statistically significant (*P* < 0.05). When PTEN is transfected with Notch1 siRNA into gastric cancer cells, the expression level of PTEN decreases. When doxorubicin is administered after transfection, the expression of PTEN increases.

## 5. Conclusions

It is well known that gastric cancer and colon cancer are highly malignant and serious wasting diseases among gastrointestinal tumors, which not only cause physical damage to the patient but also have a serious psychological impact, which seriously affects the treatment effect. Chemotherapy is an aggressive and damaging treatment process. Various adverse reactions such as anemia, reduction of granulocytes, nausea and vomiting, diarrhea, and hair loss often occur in clinical practice. It is safe and effective to perform aerobic combined resistance exercise for patients with gastrointestinal tumors after treatment. Compared with a single aerobic exercise, aerobic combined resistance exercise can bring additional benefits to patients. This study further suggests that the XPD751 gene polymorphism and common digestive system tumors may have a correlation in the Asian population. Although a certain gene polymorphism can increase or decrease the risk of cancer, the risk of an individual is not enough to be caused by its single effect. Therefore, it is necessary to carry out a multicenter study with larger sample size, broader field of view, more rigorous design, and full consideration of the environment-gene and gene-gene interaction to clarify the relationship between the two and, for the prevention, diagnosis and diagnosis of digestive system tumors. Treatment provides help.

## Figures and Tables

**Figure 1:** The influence of digestive tract microorganisms on cancer treatment.

**Figure 2:** Symptom clusters of patients with gastrointestinal cancer during chemotherapy.

**Figure 3:** Comparison of BFI scores between the two groups.

**Figure 4:** Ultrasound appearance of gastrointestinal tumors.

**Figure 5:** Comparison of weight changes of patients with different nutritional status 48 hours after admission and 7 days after operation.

**Figure 6:** Relationship between EphA1 mRNA expression and clinicopathological indicators.

**Figure 7:** RT-PCR method to detect the relative expression of PTEN and Notch1 mRNA when adriamycin interferes with gastric cancer cells BGC-823 at different time gradients.

**Table 1:** The influence of time and intervention factors on the objective nutritional indicators of the two groups of patients.

Project	Main effect of time		Main effect of intervention		Interaction effect	
	*F*	*P*	*F*	*P*	*F*	*P*
BMI	36.895	<0.001	4.268	0.045	6.584	0.003
ALB	17.599	<0.001	19.009	0.001	3.398	0.042
HB	18.359	<0.001	20.030	<0.001	3.930	0.027

**Table 2:** Performance evaluation of AdaBoost diagnostic model.

	ACC (%)	PRE (%)	REC (%)	*F*1 score (%)
Pred1	89.64	89.24	68.62	77.58
Pred2	89.05	85.79	67.72	75.69
Pred3	89.87	87.37	69.66	77.52
Pred4	90.48	89.24	70.41	78.71
Pred5	90.51	90.81	68.57	78.14

**Table 3:** Combined effect size of dual-contrast ultrasound in the diagnosis of T staging of gastric cancer.

	T1 (95% CI)	T2 (95% CI)	T3 (95% CI)	T4 (95% CI)
Sen	0.805	0.758	0.845	0.854
Spe	0.979	0.916	0.867	0.968
LR−	0.249	0.274	0.182	0.159
LR+	37.577	9.039	6.478	23.987
AUC	0.9705	0.8925	0.9283	0.9828

**Table 4:** Comparison of lower extremity vein diameter (mm) between the two groups before and after surgery.

	Grouping	External iliac vein diameter (mm)	Diameter of common femoral vein (mm)	Diameter of deep femoral vein (mm)	Popliteal vein diameter (mm)
Preoperative	IPC	9.476 ± 0.488	8.524 ± 0.127	8.948 ± 0.505	5.714 ± 0.061
	IPC + GCS	9.312 ± 1.279	8.596 ± 0.135	8.938 ± 0.490	5.720 ± 0.634

Postoperative	IPC	9.490 ± 0.486	8.538 ± 0.127	8.954 ± 0.050	5.720 ± 0.064
	IPC + GCS	9.514 ± 0.185	8.608 ± 0.144	8.942 ± 0.499	5.730 ± 0.061

**Table 5:** Comparison of the degree of total fatigue and the degree of each dimension before and after the exercise prescription intervention.

	Total fatigue score	Behavior and severity	Emotional aspect	Sensory aspect	Cognitive and emotional aspects
Before intervention	4.89 ± 1.92	5.48 ± 2.43	4.26 ± 2.38	5.41 ± 2.05	4.38 ± 2.01
Intervention for 14 days	4.32 ± 1.91	5.11 ± 2.41	3.63 ± 2.17	4.81 ± 2.26	3.69 ± 2.03
Intervention for 28 days	4.24 ± 1.97	4.86 ± 2.39	3.46 ± 2.19	4.94 ± 2.29	3.70 ± 2.23

## Data Availability

No data were used to support this study.
